The article "Association between Serum Cys C and PTB Cavitation" was published in 2023. Journal: Dis Markers.

# Association between Serum Cys C and PTB Cavitation

**DOI:** 10.1155/2023/6465182

**Published:** 2023-04-12

**Authors:** Shumin Tan, Duochi Wu, Yeying Wu, Xing Ren, Jiaxiu Liu, Xiaobin Wei

**Affiliations:** Department of Clinical Laboratory, Haikou City People's Hospital, Affiliated Haikou Hospital, Xiangya School of Medicine, Central South University, Haikou, Hainan, China

## Abstract

**Background:**

Cystatin C (Cys C) not only regulates the body's immune defenses but also contributes to tissue degradation and destruction by causing an imbalance between protease and antiprotease in infectious diseases. Is Cys C involved in pulmonary tuberculosis (PTB) infection and cavitation? We therefore conducted a retrospective study on this question to provide a basis for further studies.

**Methods:**

Cavitary PTB patients, noncavitary PTB patients, and healthy controls were recruited in our study. Serum Cys C, CRP, BUN, UA, and CR were measured in all subjects, and the Kruskal-Wallis test was used to compare medians of these clinical parameters in different groups. The Spearman rank correlation test was used to determine correlations between variables. In addition, a multivariate analysis using binary logistic regression was used to identify factors associated with PTB cavitation.

**Results:**

In our study, elevated serum Cys C levels were found in cavitary PTB patients compared to healthy controls and noncavitary patients (*p* = 0.022). Serum Cys C levels were statistically correlated with serum BUN and CR concentrations (*r* = 0.278, *p* = 0.005; *r* = 0.281, *p* = 0.004) in PTB patients. The binary logistic regression analysis showed that elevated serum Cys C levels were correlated with pulmonary cavitation in PTB patients (OR = 1.426, 95% CI: 1.071–1.898).

**Conclusion:**

Elevated serum levels of Cys C are associated with pulmonary cavitation in PTB patients.

## 1. Introduction

Pulmonary tuberculosis (PTB) is a chronic infectious disease caused by *Mycobacterium tuberculosis* (Mtb) that poses a serious public health threat [1]. Despite various public health programs and significant investments, TB remains the second leading cause of death from infectious diseases after COVID-19 and poses a major challenge to global health security [2]. PTB cavitation, a radiological hallmark of active PTB, is a severe form of tuberculosis. Studies have shown that PTB cavitation is associated with a high bacterial burden, sputum-negative conversion, and disease relapse, contributing to the high contagiousness, morbidity, and mortality of PTB [3, 4].

In the pathogenesis of PTB cavitation, the balance between protease and antiprotease plays a key role, with an MMP/TIMP imbalance being one of the typical ones [5]. Secreted by bacilli-activated innate immune cells, matrix metalloproteinase (MMP) degrades the lung extracellular matrix, whereas metalloproteinase (TIMP) inhibits this function of MMP. During the formation and development of PTB cavities, the balance of the MMPs and TIMPs interaction tips. Moreover, a growing number of studies have shown that other proteases, including cathepsin, are also involved in this complex process [6]. In addition, the activity of cathepsin is also manipulated by MTB and affects the survival of MTB in macrophages [7]. The role of cathepsin in tuberculosis has attracted increasing attention. To our surprise, cystatin C (Cys C), an inhibitor of cathepsin, has received little attention in tuberculosis research, especially in cavitary PTB.

Cys C is an endogenous cysteine protease inhibitor secreted by nucleated cells. Cys C in serum has a low molecular mass and is readily filtered through the glomerulus, making it an ideal biomarker for glomerular filtration rate (GFR) evaluation and renal function assessment [8]. In addition, serum Cys C is regulated by inflammatory cytokines, pathogens, and hormones [9]. Fluctuations in Cys C can be observed in a variety of diseases, including infections, inflammations, immune disorders, and malignancies. Recent studies also demonstrate the involvement of Cys C in tissue and elastolysis degradation through a protease/antiprotease imbalance mechanism in lung inflammation, including exacerbation of COPD and emphysema. In parasitic infections, this mechanism contributes to parasite invasion and transmission [10].

Cavity formation is routinely triggered by matrix degradation and elastolysis in low-grade inflammation during PTB development [11–13]. The question of whether Cys C is associated with pulmonary tuberculosis cavitation has piqued our interest. Therefore, we conducted this study to investigate Cys C levels in patients with cavitary tuberculosis. In addition, the associations between serum Cys C and inflammatory indicators, biomarkers of renal function, and smoking exposure were investigated. The potential role of Cys C in PTB cavitation was further explored by binary logistic regression analysis.

## 2. Materials and Methods

### 2.1. Ethical Approval

This retrospective study was conducted in the Department of Infection of Haikou City People's Hospital from August 2020 to October 2022. The protocol was approved by the ethics committee of this hospital and was conducted in accordance with the Declaration of Helsinki.

### 2.2. Study Population

A total of 103 PTB patients were enrolled in our study. The diagnosis of PTB was based on a combination of clinical symptoms, etiological examinations, chest radiologic images, and clinical laboratory tests. PTB patients were divided into cavitary and noncavitary groups based on radiological characteristics. All subjects in our study were newly diagnosed treatment-naïve cases. PTB patients who had (1) diabetes, chronic kidney diseases, emphysema, or cardiovascular diseases (including hypertension or coronary artery disease); (2) human immunodeficiency virus (HIV), hepatitis B virus (HBV), or hepatitis C virus (HCV) infection; and (3) no detailed clinical information, radiological records, and laboratory data were excluded from our study. Forty-two healthy individuals from our health centers were selected as healthy controls.

### 2.3. Clinical Record Review

The clinical data of PTB patients, including demographics (age, gender, height, weight, and BMI), clinical symptoms onset at admission, history of alcohol and smoking consumption, radiological interpretations, and laboratory measurements, were obtained in a standard format from the electronic medical record.

### 2.4. Radiological Evaluations and Clinical Laboratory Measurements

All PTB patients underwent computed tomography (CT) scans of the chest within 1 week of admission. Radiographic diagnosis of PTB and identification of cavitary PTB were performed by two experienced specialists. Any disagreements were resolved by consensus.

Sputum was collected for etiological examinations, including acid-fast bacilli staining (AFB) and M. tuberculosis culture at each patient. Blood samples were collected from all subjects after a 12-hour overnight fast using a vacuum blood collection tube without anticoagulant. An automatic analyzer measured the Cys C and other biochemical parameters (BUN, UA, Cr, and GFR) concentrations in the sera of all subjects, separated from clotted blood samples, at 3000 rpm for 10 minutes. CRP levels were measured with Mindray BC-5390. Appropriate quality assurance procedures were carried out to ensure the reliability of the measurements.

### 2.5. Statistical Analysis

In our study, continuous variables were described by medians (lower quartile and upper quartile) and analyzed by the Kruskal-Wallis test. Categorical variables were presented as ratios and compared using the Chi-square test. Correlations between variables were assessed using the Spearman rank correlation test. Furthermore, binary logistic regression analysis was done to adjust confounding factors and identify factors associated with PTB cavitation. The Statistical Package for the Social Sciences (version 26.0; SPSS, IBM, Inc.) was applied to analyze our data, and a *p* value < 0.05 was considered statistically significant. GraphPad Prism 8 (GraphPad Software, Inc.) was used to visualize the distribution of serum Cys C levels among three groups as well as the correlations between variables.

## 3. Results

The demographic characteristics of the HC, cavitary, and noncavitary PTB groups are presented in Table 1. The median age was not statistically different between the groups. The male-to-female ratio in the cavitary PTB group was higher than in the healthy control and noncavitary groups.

### 3.1. Elevated Serum Cys C in Cavitary PTB

Table 1 also describes the comparison of symptomatic episodes and CT manifestations in the cavitary and noncavitary PTB groups. Our study indicated that hemoptysis symptoms and positive staining results of acid-fasting bacilli (AFB(+)) were more common in PTB patients with cavities than in those without cavities (37.70% to 9.52%; *p* = 0.001, 29.51% to 7.14%; *p* = 0.006).

In addition, compared with HC and noncavitary PTB, the serum Cys C levels in cavitary PTB patients were higher (*p* = 0.022). There was no significant difference in serum Cys C in the comparison of noncavitary PTB with HC. The differences in CRP levels and other biochemical parameters (BUN, UA, CR, and GFR) between the HC and PTB groups were not statistically significant. The distribution of serum Cys C in the HC and PTB groups is shown in Figure 1.

### 3.2. Correlations between Serum Cys C and Renal Function Biomarkers

Correlations between serum Cys C and clinical parameters (CRP, BUN, UA, and CR) were investigated in our study. We found a fair correlation between serum Cys C level and BUN and CR in the PTB group (*r* = 0.278, *p* = 0.005^∗^; *r* = 0.278, *p* = 0.005^∗^), as shown in Figure 2. We did not find a correlation between serum Cys C and CRP. Besides, we conducted a correlation analysis between serum C and smoking exposure and did not find meaningful results.

### 3.3. Relationship between Serum Cys C and PTB Cavitation

Binary logistic regression analyses were performed to investigate the factors associated with cavitation in PTB patients (multicollinearity checks were performed, and variables with a *p* < 0.1 in Table 1 were all enrolled in the regression analyses).  Table 2 shows that a higher level of Cys C was a risk factor for PTB cavitation (OR = 1.426, 95% CI: 1.071–1.898). In addition, patients who had hemoptysis symptoms or positive AFB smears in sputum were more likely to be cavitary PTB (OR = 0.086, 95% CI: 0.021–0.344; OR = 0.067, 95% CI: 0.013–0.342).

## 4. Discussion

In the present study, elevated serum Cys C levels were found in cavitary PTB patients compared to healthy controls and noncavitary PTB patients. Serum Cys C correlated with serum BUN and CR in PTB. Binary logistic regression analysis indicated that serum Cys C was correlated with PTB cavitation.

Cys C is a small, low-molecular-weight protein secreted by almost all nucleated cells, freely filtered by the glomerular membrane, and then completely absorbed by the proximal tubular cells without being secreted. This property makes serum Cys C a promising indicator of renal function, like serum urea and creatine [8, 14]. Furthermore, as an innate endogenous cathepsin inhibitor, Cys C is involved in tissue destruction by upsetting the balance between Cys C and cathepsin. A growing number of studies have shown that Cys C also regulates the body's immune function at both molecular and cellular levels [9]. In turn, the secretion of Cys C is also regulated by multiple cytokines or pathogenic bacteria [10]. Considering its position in the complex network of immune regulation, Cys C plays a key role in the development and progression of disease, not merely as a marker of renal function.

PTB cavitation is a severe form of tuberculosis characterized by the degradation of lung tissue. Not only does PTB cavitation severely affect patients' respiratory function but it is also associated with the spread and persistence of PTB. In the pathology of PTB cavitation, the host immune response and the protease/antiprotease balance play a pivotal role. One of the most widely investigated is MMP, a matrix-degrading protease secreted by monocyte-derived cells and neutrophils and tightly regulated in our body. Elevated MMP levels in serum and lung tissue have been found in cavitary PTB patients. The imbalance between MMP and its inhibitor drives cavity formation [5, 12, 13]. A recent transcriptomic study performed in a rabbit cavitary PTB model identified that multiple proteases, including MMP and cathepsin, are upregulated during PTB cavitation [6]. Similar to MMP, cathepsin is exerted during extracellular matrix degradation to facilitate PTB invasion and transmission. In turn, this function of cathepsin can be regulated by Cys C, an endogenous antiprotease specific to cathepsin. Anomalous cathepsin expression in cavitary PTB has been identified in several investigations, but there have been few studies involving Cys C. Elevated serum Cys C has been found in some inflammatory pulmonary diseases with tissue degradation [15, 16]. However, in the related field of tuberculosis, Cys C has been studied mainly as a predictor of renal impairment during antituberculosis drug therapy or to predict the risk of complications of tuberculosis [17–19]. To the best of our knowledge, our study is the first to explore the relationship between serum Cys C and PTB cavitation in clinic.

As shown in Figure 1, we did not find any significant difference in serum Cys C levels between noncavitary PTB patients and healthy controls. Elevated serum Cys C levels were found in cavitary PTB patients compared to healthy controls and noncavitary patients. Wu et al. reported that serum Cys C concentrations did not differ between PTB patients and healthy controls. Elevated serum Cys C levels were observed only in PTB patients with comorbid chronic diseases. Regrettably, the PTB patients in their study were not divided into cavitary or noncavitary groups [19]. Together, these studies suggest that the association of elevated serum Cys C with tuberculosis is evident in the cavitary PTB group, characterized by lung tissue degradation. A previous study has demonstrated that upregulated expression of cathepsin is related to the occurrence of pulmonary cavitation [6]. It is reasonable to speculate that the elevated serum Cys C in PTB cavitation may be a compensatory reaction after matrix degradation induced by cathepsin, which plays a role in lung tissue degradation and cavity formation. In addition, the clinical characteristics of cavitary PTB patients are shown in Table 1. We discovered that AFB(+) and hemoptysis were more common in PTB patients with cavities than in those without cavities. After adjustment for confounding factors, this association persisted (Table 2), indicating that cavitary PTB patients have a higher MTB load and blood vessel rupture. Therefore, we speculate that Cys C may participate in PTB cavitation via additional mechanisms. Recent studies have shown that Cys C plays a crucial role in regulating antigen presentation, protecting the host from microbial invasion, and inhibiting viral replication and growth [20–23]. Elevated Cys C levels associated with high viral loads have been found in HIV patients [24]. We boldly hypothesized that elevated serum Cys C might be a function of the immune defense against the high load of Mtb in cavitary PTB. In addition, PTB cavitation is more likely to invade blood vessels and cause hemoptysis symptoms. A previous study demonstrated that elevated serum Cys C levels may be involved in cognitive dysfunction caused by cerebral microbleeds in cerebral hemorrhage patients [25]. Another study has shown that Cys C plays an essential role in the vascular remodeling of damaged arteries [26]. Therefore, we speculate that vascular injury and remodeling in PTB cavitation may be responsible for elevated serum Cys C. Regrettably, due to the small samples in our study, further analysis of the correlation between hemoptysis or bacterial load and Cys C in cavitary PTB is not appropriate. Further in-depth studies incorporating more subjects are required to test our conjectures.

As shown in Figure 2, serum Cys C correlated with serum BUN and CR in PTB, suggesting the prospect of serum Cys C as a biomarker of renal function to some extent in accordance with a previous study [15]. Another study has also shown that Cys C is an indicator of kidney injury associated with antituberculosis drugs [17]. It is certain that serum Cys C is affected by renal function and interferes with the experimental result interpretation in our study. Given these considerations, when investigating the relationship between serum Cys C and PTB cavitation, we adjust the confounding factors (including BUN and CR) using binary logistic regression analysis to improve the accuracy and reliability of our findings. As shown in Table 2, serum Cys C is closely associated with PTB. The higher the serum Cys C levels, the greater the likelihood of lung cavitation in PTB patients.

Considering the effect of antituberculosis therapy on serum Cys C levels, we recruited treatment-naïve PTB patients to participate in our study [17]. To explore the relationship between serum Cys C and PTB cavitation, we used binary logistic regression analysis to adjust for the effects of multiple confounding factors and make our results more accurate. There were some limitations in our study. First and foremost, this was a small sample size study, limiting future research on Cys C and clinical symptoms in cavitary PTB. Second, Cys C was only measured in serum; we did not measure its concentration in lavage fluid or lung tissue. In addition, we did not measure both cathepsin and other lung tissue degradation indicators such as MMPs. Therefore, more in-depth and considered investigations will be required in the future.

## 5. Conclusion

Elevated serum levels of Cys C are associated with pulmonary cavitation in PTB patients.

## Figures and Tables

**Figure 1:** Elevated serum Cys C in cavitary PTB. Elevated serum Cys C levels were found in patients with cavitary PTB compared to noncavitary PTB and healthy controls. Serum Cys C concentrations were measured in 61 cavitary PTB patients, 42 noncavitary PTB patients, and 42 healthy controls. Lines and whiskers represent median and interquartile values. Data were analyzed by Kruskal Wallis test with Dunn's multiple comparisons. Statistically significant differences are highlighted. ^∗^*p* < 0.05. Cys C: cystatin C; PTB: pulmonary tuberculosis; HC: healthy controls.

**Figure 2:** Correlation between serum Cys C and renal function parameters in PTB. (a) Serum Cys C was positively correlated with serum BUN. (b) Serum Cys C was positively correlated with serum CR in PTB group. Spearman's correlation coefficient and *p* value are noted in the top left corner of the figure, ^∗^ means statistically significant. Cys C: cystatin C; PTB: pulmonary tuberculosis; BUN: blood urea nitrogen; CR: creatine.

**Table 1:** Characteristics of the three groups.

	Noncavitary PTB (*N* = 42)	Cavitary PTB (*N* = 61)	HC (*N* = 42)	*p* value
Gender (M/F)	22/20	46/15^ab^	23/19	0.026^∗^
Age (years)	31 (22.75–38.5)	36 (28–55.5)	35.5 (29–44.25)	0.085
BMI (kg/m^2^)	18.80 (17.70–21.25)	18.47 (17.19–19.98)	NA	0.457
Current/ex/never smoking	11/2/29	29/3/29	NA	0.084
Current/ex/never drinking	21/1/20	34/2/25	NA	0.789
Onset of symptoms				
Cough, number (%)	80.95%	88.52%	NA	0.284
Hemoptysis, number (%)	9.52%	37.70%^b^	NA	0.001^∗^
Sweat, number (%)	28.57%	24.59%	NA	0.652
Fever, number (%)	33.33%	22.95%	NA	0.244
CT findings				
Both lung lesions, number (%)	66.67%	72.13%	NA	0.552
Pleural thickening, number (%)	54.76%	49.18%	NA	0.578
Clinical laboratory tests				
Sputum positive, number (%)	7.14%	29.51%^b^	NA	0.006^∗^
CRP (ng/L)	21.74 (8.54–71.11)	14.93 (2.48–57.07)	NA	0.167
Cys C (mg/L)	0.79 (0.67–0.88)	0.87 (0.72–0.96)^ab^	0.79 (0.74–0.83)	0.022^∗^
BUN (mmol/L)	3.55 (2.80–4.46)	3.87 (3.09–4.61)	4.28 (3.50–4.81)	0.091
UA (umol/L)	305.50 (242.75–356.75)	301.00 (247.00–365.00)	307.00 (255.25–347.50)	0.984
CR (umol/L)	61.00 (54.50–70.00)	68.00 (57.50–76.00)	67.00 (55.00–76.00)	0.078
GFR (ml/min)	128.00 (118.00–144.00)	126.23 (109.00–140.00)	116.00 (106.00–137.00)	0.076

BMI: body mass index; CRP: C-reactive protein; Cys C: cystatin C; BUN: blood urea nitrogen; UA: uric acid; CR: creatine; GFR: glomerular filtration rate; NA: not available. ^∗^*p* < 0.05; statistic significant (Kruskal-Wallis test with Dunn multiple test comparison or Chi-square test); ^a^*p* < 0.05, compared with healthy control; ^b^*p* < 0.05, compared with noncavitary PTB.

**Table 2:** Factors associated with PTB cavitation.

Variable	*b*	*S*_*b*_	Wald *X*^2^	*p*	OR	95% CI
Gender	-0.621	0.790	0.617	0.432	0.537	0.114–2.530
Hemoptysis	-2.453	0.707	12.033	0.001^∗^	0.086	0.021–0.344
AFB (+)	-2.701	0.831	10.572	0.001^∗^	0.067	0.013–0.342
BUN	0.127	0.221	0.330	0.566	1.135	0.737–1.749
CR	0.008	0.031	0.061	0.804	1.008	0.949–1.070
Cys C	0.355	0.146	5.912	0.015^∗^	1.426	1.071–1.898
Smoking history						
Current smoking (1)	0.053	0.649	0.007	0.935	1.054	0.295–3.762
Ex smoking (2)	-1.503	1.208	1.550	0.213	0.222	0.021–2.371

Binary logistic regression analyses were performed to adjust confounding factors and evaluate the factors associated with PTB cavitation. AFB(+): positive result of acid-fasting bacilli staining; BUN: blood urea nitrogen; Cys C: cystatin C; CI: confidence interval; ^∗^*p* < 0.05, statistic significant.

## Data Availability

The datasets used and/or analyzed during the current study are available from the corresponding author on reasonable request.
